RETRACTED

# Optimized Turmeric Extract Reduces β-Amyloid and Phosphorylated Tau Protein Burden in Alzheimer’s Transgenic Mice

**DOI:** 10.2174/156720512800492459

**Published:** 2012-05

**Authors:** R Douglas Shytle, Jun Tan, Paula C Bickford, Kavon Rezai-zadeh, L Hou, Jin Zeng, Paul R Sanberg, Cyndy D Sanberg, Randall S Alberte, Ryan C Fink, Bill Roschek

**Affiliations:** a Center for Excellence in Aging and Brain Repair, Dept. of Neurosurgery; b Silver Child Development Center, Dept. of Psychiatry and Behavioral Medicine; c Neuroscience Program, University of South Florida College of Medicine, Tampa, FL 33612; d Veterans Administration Hospital, Research Service, Tampa, FL 33612; e Natura Therapeutics, Inc, 3802 Spectrum Blvd, Tampa, FL 33612; f deceased: October 4, 2010; g Department of Food Science and Nutrition, University of Minnesota, St. Paul, MN 55108; h HerbalScience Group LLC., Naples, FL 34110, USA

**Keywords:** Alzheimer’s disease, Tau phosphorylation, turmeric, curcuminoids.

## Abstract

In a previous *in vitro* study, the standardized turmeric extract, HSS-888, showed strong inhibition of Aβ aggregation and secretion *in vitro*, indicating that HSS-888 might be therapeutically important. Therefore, in the present study, HSS-888 was evaluated *in vivo* using transgenic ‘Alzheimer’ mice (Tg2576) over-expressing Aβ protein. Following a six-month prevention period where mice received extract HSS-888 (5mg/mouse/day), tetrahydrocurcumin (THC) or a control through ingestion of customized animal feed pellets (0.1% w/w treatment), HSS-888 significantly reduced brain levels of soluble (~40%) and insoluble (~20%) Aβ as well as phosphorylated Tau protein (~80%). In addition, primary cultures of microglia from these mice showed increased expression of the cytokines IL-4 and IL-2. In contrast, THC treatment only weakly reduced phosphorylated Tau protein and failed to significantly alter plaque burden and cytokine expression. The findings reveal that the optimized turmeric extract HSS-888 represents an important step in botanical based therapies for Alzheimer’s disease by inhibiting or improving plaque burden, Tau phosphorylation, and microglial inflammation leading to neuronal toxicity.

## INTRODUCTION

Alzheimer's Disease (AD) is characterized by intra- and extracellular lesions known as neurofibrillary tangles and amyloid plaques respectively. The neuropathological diagnosis of AD can be determined only post-mortem and requires the presence of both senile plaques and neurofibrillary tangles (NFT) [1]. Senile plaques are largely composed of amyloid-β (Aβ) peptides, whereas NFTs are composed of hyperphosphorylated Tau protein organized into paired helical filaments [2-4].

RETRACTED

The central theme of the current Aβ cascade hypothesis is the accumulation in the brain of Aβ initiating a series of pathological reactions causing chronic inflammation [5]. These conditions lead to Tau aggregation and neuronal dysfunction, the primary causes of dementia [6]. The accumulation of Aβ results from the secretase driven cleavage product of the amyloid precursor protein (APP), both as soluble aggregate oligomers and insoluble fractions associated with senile plaques.

The formation of NFTs has gained center stage as a cause of the pathology associated with AD. Tau is a group of microtubule-associated proteins expressed predominantly in axons [7, 8]. Hyperphosphorylated Tau is observed in the developing fetal brain and in the AD brain [9-12]. In both cases, some neurons are degenerating, suggesting that the phosphorylation of Tau may directly or indirectly play a part in neuronal cell death through the destabilization of microtubules.

The number of therapeutic treatments for AD is limited with pharmaceuticals available currently approved for the treatment of symptoms only and not prevention of the disease [13, 14]. In addition, many promising drug candidates fail in clinical trials for reasons unrelated to their efficacy [14] and drug discovery using synthetic methodologies is expensive and inefficient [15]. Our research group and others have therefore been focusing on the screening of botanical extracts where therapeutic benefits have been documented by traditional medicine systems [16, 17].

Curcumin (diferuloylmethane; Cur) is an orange-yellow component of the curry spice turmeric (*Curcuma longa *L.). Traditionally known for its anti-inflammatory effects, Cur has been shown to be a potent therapeutic agent with reported beneficial effects for asthma, arthritis, atherosclerosis, cancer, and diabetes [18-22]. Additional *in vitro* results have shown that Cur attenuates inflammatory activation of microglial cells, prevents neuronal damage, and reduces oxidative damage in the brain [23-29]. 

In a previous study by our group [30], we compared the efficacy of three proprietary turmeric extracts (HSS-888, HSS-838, and HSS-848), each having different chemical profiles and relative abundances of the different curcuminoids and turmerones, with various curcuminoid standards: Cur, DMC (Demthoxycurcumin), BDMC (Bisdemethoxycurcumin), and THC. All three extracts and the curcuminoids showed dose-dependent inhibition of Aβ aggregation from Aβ_1-42 _in a cell-free assay with IC_50_ values of <5 μg/mL. However, only HSS-888, Cur and DMC significantly decreased Aβ secretion (~20%) in SweAPP N2A cells [30]. Because HSS-888 showed strong inhibition of Aβ aggregation and secretion, this extract was utilized in the present *in vivo* study using transgenic a transgenic mouse model for AD (Tg2576 mice) that over-express Aβ protein in order to determine the pathological response of Aβ aggregation and Tau phosphorylation when an optimized turmeric extract was consumed.

RETRACTED

## MATERIALS AND METHODS

### Turmeric Extracts and Reagents

A standardized turmeric (*Curcuma longa* L.) extract, HSS-888, was prepared using proprietary supercritical CO_2_ extraction methods (HerbalScience Singapore Pte Ltd). Extract HSS-888 contains 82% curcuminoids by weight. Tetrahydrocurcumin (THC) was obtained from Chromadex (Irvine, CA) and was about 40% pure THC and about 60% of a reduced form of THC [30].

Anti-human amyloid-β antibodies 4G8 and 6E10 were obtained from Signet Laboratories (Dedham, MA) and Biosource International (Camarillo, CA), respectively. VectaStain Elite™ ABC kit was obtained from Vector Laboratories (Burlingame, CA). Aβ_1-40, 42 _ELISA kits were obtained from IBL-American (Minneapolis, MN). Anti-phospho-Tau antibodies including Ser^199/220^ and AT8 were purchased from Innogenetics (Alpharetta, GA).

### *In Vivo* Treatment

The Tg2576 mice were purchased from Taconic (Germantown, NY). For oral administration of extracts, a total of 60 (30 female/30 male) Tg2576 mice with a B6/SJL background were employed. Beginning at 8 months of age, Tg2576 treatment mice were administered the optimized turmeric extract HSS-888 (0.1% w/w) or THC (0.1% w/w) in NIH31 chow or NIH31 chow alone (Control) for 6 months [n = 20 (10 female/10 male)]. All mice were sacrificed at 14 months of age for analyses of Aβ levels and Aβ load in the brain according to previously described methods [31]. Animals were housed and maintained in the College of Medicine Animal Facility at the University of South Florida (USF), and all experiments were in compliance with protocols approved by the USF Institutional Animal Care and Use Committee.

### Immunohistochemistry

Mice were anesthetized with isofluorane and transcardially perfused with ice-cold physiological saline containing heparin (10 U/mL). Brains were rapidly isolated and quartered using a mouse brain slicer (Muromachi Kikai Co., Tokyo, Japan). The first and second anterior quarters were homogenized for ELISA and Western blot analysis as described below, and the third and fourth posterior quarters were used for microtome or cryostat sectioning. Brains were then fixed in 4% (w/v) paraformaldehyde in PBS at 4°C overnight and routinely processed in paraffin in a core facility at the Department of Pathology (USF College of Medicine). Five serial coronal sections (5 µm) spaced ~150 µm apart from each brain section were selected for immunohistochemical staining and image analysis. Sections were routinely deparaffinized and hydrated in a graded series of USP ethanol prior to pre-blocking for 30 min at ambient temperature with serum-free protein block (Dakocytomation, Glostrup, Denmark). The Aβ immunohistochemical staining was performed using anti-human β-antibody (clone 4G8, 1:100) in conjunction with the VectaStain Elite™ ABC kit coupled with diaminobenzidine substrate. The 4G8-positive Aβ deposits were examined under bright-field using an Olympus BX-51 microscope. Quantitative image analysis (conventional “Aβ burden” analysis) was routinely performed for 4G8 immuno-histochemistry. Data are reported as percentage of immunolabeled area captured (positive pixels) divided by the full area captured (total pixels). 

RETRACTED

### Image Analysis

Quantitative image analysis (conventional “Aβ burden” analysis) was performed using stereological methods for 4G8 immuno-histochemistry and Congo red histochemistry for brains from Tg2576 mice orally administrated THC, HSS-888, or NIH31 control chow. Images were obtained using an Olympus BX-51 microscope and digitized using an attached MagnaFire™ imaging system (Olympus, Tokyo, Japan). Briefly, images from five serial sections (5 µm) spaced ~150 µm apart through each anatomic region of interest (hippocampus or cortical areas) were captured and a threshold optical density was obtained that discriminated staining form background. Manual editing of each field was used to eliminate artifacts. Data are reported as percentage of immunolabeled area captured (positive pixels) divided by the full area captured (total pixels). Quantitative image analysis was performed by a single examiner blinded to sample identities. 

### Aβ ELISA

Mouse brains were isolated under sterile conditions on ice and placed in ice-cold lysis buffer (20 mM Tris, pH 7.5, 150 mM NaCl, 1mM EDTA, 1 mM EGTA, 1% [v/v] Triton X-100, 2.5 mM sodium pyrophosphate, 1 mM β-glycerol-phosphate, 1 mM Na_3_VO_4_, 1 µg/mL leupeptin, 1 mM PMSF) as previously described [32]. Brains were then sonicated on ice for approximately 3 min, allowed to stand for 15 min at 4°C, and centrifuged at 15,000 rpm for 15 min. Insoluble Aβ_1-40, 42_ species were detected by acid extraction of brain homogenates in 5 M guanidine buffer [33], followed by a 1:10 dilution in lysis buffer. Soluble Aβ_1-40, 42_ were directly detected in brain homogenates prepared with lysis buffer described above by a 1:10 dilution. Protein levels of homogenate samples were all normalized by BCA protein assay prior to dilution. Aβ_1-40, 42 _was quantified using an Immuno-Biological Laboratories non-discriminate Aβ ELISA kit in accordance with the manufacturer’s instructions, except that standards included 0.5 M guanidine buffer in some cases. 

RETRACTED

### Western Blot Analysis

Brain homogenates were obtained as previously described above. For Tau analysis, aliquots corresponding to 100µg of total protein were separated electrophoretically using 10% Tris gels. Electrophoresed proteins were then transferred to nitrocellulose membranes (Bio-Rad, Richmond, CA), washed in ddH_2_O, and blocked for 1 h at ambient temperature in Tris-buffered saline (TBS) containing 5% (w/v) non-fat dry milk. After blocking, membranes were hybridized for 1 h at ambient temperature with various primary antibodies. Membranes were then washed 3 times for 5 min each in ddH_2_O and incubated for 1 h at ambient temperature with the appropriate HRP-conjugated secondary antibody (1:1,000, Pierce Biotechnology, Woburn, MA). All antibodies were diluted in TBS containing 5% (w/v) of non-fat dry milk. Blots were developed using the Luminol reagent (Pierce Biotechnology, Woburn, MA). Densitometric analysis was done as previously described using a FluorS Multiimager with Quantity One™ software (BioRad, Hercules, CA) [34]. 

### Cytokine ELISA

As described in previous studies [35, 36], cell cultured microglia were collected for measurement of cytokines by commercial cytokine ELISA kits. In parallel, cell lysates were prepared for measurement of total cellular protein. Data are represented as ng/mg total cellular protein for each cytokine produced. Cytokines were quantified using commercially available ELISAs (BioSource International, Inc., Camarillo, CA) that allow for detection of IL-2 and IL-4. 

### Statistical Analysis

All data were normally distributed; therefore, Levene’s test for equality of variances, followed by *t*-test for independent samples, was used to assess significance in instances of single mean comparisons. Single Factor ANOVA analysis was used for between group variations when multiple groups were combined using Microsoft Excel Data Analysis Tools. The statistical package for the social sciences release 10.0.5 (SPSS Inc., Chicago, IL) or Statistica^©^ were used for all other data analyses.

## RESULTS

### Oral Administration of HSS-888 Reduces Cerebral Amyloidosis

We recently demonstrated that the optimized turmeric extract HSS-888 is an effective inhibitor of both Aβ secretion and aggregation *in vitro *[30]. To determine whether oral administration of this extract could have similar anti-amyloidogenic effects *in vivo*, 8-month old Tg2576 mice were fed an HSS-888 supplemented, THC supplemented, or control diet for a period of 6 months. As shown in Fig. (**1A**), HSS-888 treatment reduced Aβ deposition in these mice compared to both control and THC treatments. Image analysis of micrographs from Aβ antibody (4G8) stained sections revealed that plaque burdens were significantly reduced throughout the entorhinal cortex (EC, 5.9% plaque burden; *P*<0.01) and hippocampus (H, 1.8%;* P*<0.05) compared to control plaque burdens of 8.9% and 3.5% for the EC and H respectively Fig. (**1**). 

RETRACTED

To verify the findings from these coronal sections, we analyzed brain homogenates for Aβ levels by ELISA. Again, oral treatment of HSS-888, significantly reduced soluble (1640 pg/mg; *P*<0.05) and insoluble (4310 pg/mg; *P*<0.05) forms of Aβ_1-40, 42 _compared to soluble (2850 pg/mg) and insoluble (4910 pg/mg) controls Fig. (**2**). THC did not significantly reduce either soluble or insoluble of Aβ_1-40, 42_. Collectively, the above data confirms that orally administered HSS-888 provides effective attenuation of amyloid deposition. 

It should be noted that the THC used here was approximately 40% THC and 60% a reduced form of THC. Based on our previous experiments showing pure THC increases Aβ production [30], it can be reasonably concluded from these results that reduced THC may afford some protection from Aβ production and deposition compared to the non-reduced form. This protection is minimal compared to HSS-888.

### Oral Administration of HSS-888 Reduces Tau Hyperphosphorylation 

To investigate the possibility that HSS-888 may also affect Tau physiology, we analyzed anterior quarter brain homogenates from the treated mice by Western blot analysis. Fig. (**3**) shows the soluble fractions of phosphorylated Tau (pTau) detected in the homogenates of the treatment groups and their control mice by both Ser^199/220^ and AT8 antibodies Fig. (**3A**). Mice treated with THC showed a 47% decrease in the ratio of pTau to Actin (0.44; *P*<0.001) relative to control (0.83). Mice treated with HSS-888 however showed an 80% decrease in pTau to Actin (0.17; *P*<0.001) relative to control mice Fig. (**3B**). 

### Oral Administration of HSS-888 Enhances Th2 Cellular Immunity

As previous studies have established the ability of Cur to both suppress an inflammatory immune response and promote the shift from Th1 to Th2 immunity [37], we investigated the ability of HSS-888 and THC to mediate these effects in Tg2576 mice. Following sacrifice of both treatment and control groups, primary cultures of microglia were established from these mice and stimulated for 24 h with anti-CD3 antibody. As illustrated in Fig. (**4**), cytokines IL-4 and IL-2 were increased to 143 ng/mg and 129 ng/mg respectively. This represents a 3-fold increase in IL-4 production and a 2-fold increase in IL-2 production compared to controls when treated with HSS-888 Fig. (**4A**). The ratio of IL-4 to IL-2 improved from 0.73 (control) to 1.11 (HSS-888; *P*<0.001; Fig. (**4B**)) indicating HSS-888 may afford microglia protection via the anti-inflammatory activity of specific cytokines.

RETRACTED

## DISCUSSION

The present study shows that an optimized turmeric extract, HSS-888, significantly reduces brain levels of soluble (~40%) and insoluble (~20%) Aβ as well as hyperphosphorylated Tau protein (~80%) in Tg2576 mice that received HSS-888 the optimized turmeric extract via customized animal feed pellets daily for six months. Furthermore, primary cultures of microglia from these mice exhibited enhanced cellular immunity (increased IL-4 to IL-2 ratio). The current *in vivo* results confirm our previous *in vitro* findings with turmeric extract HSS-888 [30].

Previous studies have suggested that soluble hyperphosphorylated isoforms are ultimately the neurotoxic species of Tau [38, 39]. Both the optimized turmeric extract (HSS-888) and THC may afford protection from the effects of these toxic Tau isoforms. HSS-888 may also provide site specific inhibition of Tau phosphorylation due to its reduction of phosphorylation detected by the AT8 antibody compared to phosphorylation detected at Ser 199/220. To our knowledge, this is the first demonstration of turmeric having *in vivo* efficacy against Tau hyperphosphorylation.

Administration of THC also decreased Tau hyperphosphroylation in the present study, however it was less effective than HSS-888 and failed to significantly affect other therapeutic endpoints such as Aβ accumulation, plaque burden, and cytokine expression. These findings are consistent with our previous *in vitro* study where THC increased Aβ accumulation in N2A cells [30]. In addition, Begum *et al.* [29] fed Cur and THC (~1.25 mg/kg/day) to aged Tg2576 APPsw mice for four months and found that only Cur re-duced amyloid plaque burden and insoluble Aβ levels in the brain. 

HSS-888 increases the production of the anti-inflammatory cytokine IL-4 in cultured microglia from HSS-888 treated mice. IL-4 is a well known anti-inflammatory cytokine known to reduce the production of inflammation mediators in microglia such as TNF-α and MCP-1 [40]. Lyons *et al.* have shown that IL-4 inhibits microglia activation and subsequent inflammation induced by Aβ [41]. Additionally, Kiyoto *et al.* showed that sustained expression of IL-4 reduces Aβ oligomerization and deposition and improves neurogenesis [42]. This data indicates that HSS-888 is also likely reducing inflammation and neuronal cell death via IL-4 production. This increase in IL-4 also likely assists with the clearance of Aβ *in vivo*, reducing neurotoxicity.

RETRACTED

HSS-888 effectively attenuates three primary mechanisms of Alzheimer’s progression. Specifically, HSS-888: 1.) reduces plaque burden in the entorhinal cortex and hippocampus; 2.) reduces Tau phosphorylation; and 3.) increases IL-4 production. Collectively, these results indicate that the turmeric extract HSS-888 contributes to the mitigation of AD pathologies *in vivo* through both direct and indirect effects on Aβ aggregation and deposition and neuronal cell protection through anti-inflammatory routes. 

## Figures and Tables

**Fig. (1):** Oral Administration of HSS-888 Results in Reducing Cerebral Amyloidosis in Tg2576 mice. (**A**) Mouse brain coronal frozen sections were stained with rabbit polyclonal anti-human Aβ antibody. The middle panel shows HSS-888-treated and the bottom panel shows THC-treated Tg2576 mice, while the top panel represents controls animals who received animal chow with no extract or THC. (**B**) Percentages of Aβ antibody-immunoreactive Aβ plaque (mean ± SD) were calculated by quantitative image analysis (n = 20). One-way ANOVA revealed significant differences (**P<0.001; *P<0.001) between groups for each brain region examined as indicated. The abbreviations are defined as follows: cingulated cortex (CC), hippocampus (H), entorhinal cortex (EC).

**Fig. (2):** Oral Treatment of HSS-888 Reduces Both Soluble and Insoluble Aβ_1-40, 42_ Levels in Mouse Brain Homogenates. (**A**) Brain homogenates prepared from Tg2576 mice treated with animal pellets only (control), HSS-888, or THC. H20 soluble Aβ_1-40, 42_ were analyzed by ELISA. (**B**) Insoluble Aβ_1-40, 42_ prepared with 5 M guanidine were analyzed by ELISA. Data are presented as mean ± SD of Aβ_1-40_ or Aβ_1-42_ (pg/mg protein) separately. For (**A**) and (**B**), a *t*-test revealed a significant between-groups difference for either soluble or insoluble Aβ_1-40, 42_ (*P* < 0.05 for each comparison) as indicated. Mean ± standard deviation for each group [n = 20 (10 male/10 female) for Controltreated, HSS-888-treated, and THC-treated Tg2576 mice].

**Fig. (3):** Tg2576 mice orally treated with HSS-888 or THC Show Decreased Phosphorylated Tau Protein. Brain homogenates were prepared from Tg2576 mice treated with Control, HSS-888 or THC. (**A**) Western blot analysis by antibody Ser^199/220^ or AT8 shows phosphorylated Tau protein as indicated. (**B**) Densitometry analysis shows the ratios of phospho-Tau AT8 to Actin band density. A *t*-test revealed a significant difference between HSS-888, or THC treatment and Control (**P < 0.001). Mean ± standard deviation for each group (n = 20 for each group).

RETRACTED

**Fig. (4):** Tg2576 Mice Orally Treated with HSS-888 Show Enhanced Th2 Cellular Immune Responses *Ex Vivo*. Primary cultures of microglia were established from these mice, and these cultures were stimulated for 24 hours with anti-CD3 antibody (mitogen,1 µg/mL). Cytokines in cultured media were measured by ELISA kits. Data were represented as pg of each cytokine per total intracellular protein (mg). A t-test revealed a significant difference for the ratio of IL-4 to IL-2 between HSS-888 and Control (**P < 0.001). Mean ± standard deviation for each group (n = 10 for each group).
